The article "Use of Multiple Doses of Intravenous Infusion of Umbilical Cord-Mesenchymal Stem Cells for the Treatment of Adult Patients with Severe COVID-19-Related Acute Respiratory Distress Syndrome: Literature Review" was published in 2023. Journal: Stem Cells Int.

# Use of Multiple Doses of Intravenous Infusion of Umbilical Cord-Mesenchymal Stem Cells for the Treatment of Adult Patients with Severe COVID-19-Related Acute Respiratory Distress Syndrome: Literature Review

**DOI:** 10.1155/2023/7179592

**Published:** 2023-08-18

**Authors:** Po-Ren Hsueh, Sung-Jung Ho, Po-Chuen Hsieh, I-Min Liu, Shio-Shin Jean

**Affiliations:** ^1^Departments of Laboratory Medicine and Internal Medicine, China Medical University Hospital, China Medical University, Taichung, Taiwan; ^2^School of Medicine, China Medical University, Taichung, Taiwan; ^3^Departments of Laboratory Medicine and Internal Medicine, National Taiwan University Hospital, National Taiwan University College of Medicine, Taipei, Taiwan; ^4^Division of Pulmonary Medicine, Department of Internal Medicine, Min-Sheng General Hospital, Taoyuan, Taiwan; ^5^Department of Pharmacy, College of Pharmacy and Health Care, Tajen University, Pingtung, Taiwan; ^6^Departments of Internal Medicine and Critical Care Medicine, Min-Sheng General Hospital, Taoyuan, Taiwan

## Abstract

**Objectives:**

Acute respiratory distress syndrome (ARDS) is a critical complication in severe COVID-19 patients. The intravenous infusion (IVF) of umbilical cord- (UC-) mesenchymal stem cells (MSCs), validated to substantially reduce the release of several inflammatory cytokines *in vivo*, was also shown to exhibit benefits in improving hypoxemia among severe COVID-19 patients. A single dose of IVF-UC-MSCs therapy for severe COVID-19 patients was shown to alleviate the initial ARDS severity, but have 50%–67% case-fatality rates. In Taiwan, few adult patients with severe COVID-19-induced ARDS receiving compassionate adjuvant treatment consisting of either a single dose (1–10 × 10^6^ cells/kg body weight (kg BW)) or three doses (5 × 10^6^ cells/kg BW in each dose) of IVF-UC-MSCs had good outcomes. However, the optimal dosage and rounds of IVF-UC-MSCs administration for the treatment of severe COVID-19 patients with ARDS are undetermined.

**Methods:**

We reviewed the 2020–2022 PubMed literature database concerning the clinical efficacy of IVF-UC-MSCs among severe COVID-19 patients.

**Results:**

The data of COVID-19 case series in the PubMed literature revealed a notable heterogeneity in the therapeutic dosage (a single dose: 1–10 × 10^6^ cells/kg BW; and three doses: 50–200 × 10^6^ cells/kg BW in each dose) and the post-ARDS days of IVF-UC-MSCs administration (a single dose: 1–12; and multiple doses: 5–14) for the treatment of severe COVID-19-associated ARDS. The survival rates among these severe COVID-19 patients ranged from 50% to 76%. However, an overall rate of 93.1% of significant improvement in hypoxemia was observed for the COVID-19 survivors receiving IVF-UC-MSCs at the initial ARDS stage.

The article "Use of Multiple Doses of Intravenous Infusion of Umbilical Cord-Mesenchymal Stem Cells for the Treatment of Adult Patients with Severe COVID-19-Related Acute Respiratory Distress Syndrome: Literature Review" was published in 2023. Journal: Stem Cells Int.

**Conclusions:**

According to our analysis, the ideal treatment dosage of IVF-UC-MSCs for severe COVID-19-induced ARDS is likely 5 × 10^6^ cells/kg BW for three cycles within 5 days of ARDS onset in severe COVID-19 patients.

## 1. Introduction

Severe respiratory syndrome coronavirus 2 (SARS-CoV-2), the main virus responsible for the coronavirus disease 2019 (COVID-19), has infected more than 760 million people around the world as of April 2023 and has also resulted in overwhelming morbidity, with more than 6 million fatalities worldwide. According to the brief review addressed by Tzotzos et al. [1] acute respiratory distress syndrome (ARDS) developed in 47%–100% of the COVID-19 patients hospitalized in the intensive care unit (ICU), and mortality rates reportedly ranged from 13% to 89% among COVID-19 patients with ARDS. To effectively manage ARDS-related hypoxemia in severe COVID-19 patients, all ICU physicians adopt aggressive strategies of the respiratory support (using ventilator mostly, or high-flow nasal canula that generates positive airway pressure instead) [2, 3]. Although prescription of dexamethasone in combination with tocilizumab [4, 5] and/or baricitinib [6] have been formally recommended to improve the survival of patients with severe COVID-19, related lung inflammation with subsequent dysfunction likely persists.

Russell et al. [7] and Biswas et al. [8] observed that COVID-19 patients with old age (age ≥ 50 years old) [7], or with a single or multiple comorbidities (including morbid obesity, hypertension, diabetes mellitus (DM), chronic pulmonary disease adversely affecting respiration, cerebrovascular disease, chronic kidney disorder, chronic human immunodeficiency virus infection with receipt of antiretroviral agent therapy, malignancy, or immunocompromised diseases related to use of various immunosuppressants etc.) had significantly increased risk of mortality [7, 8]. In-hospital complications associated with vital organ support and organ function monitor (e.g., therapy of dexamethasone, and tocilizumab/baricitinib for alleviating lung inflammation and cytokine storm, and insertions of intravenous and/or foley catheters etc.) and prolonged critical illness (e.g., corticosteroid and/or neuromuscular antagonist-related neuropathy or myopathy, or immunosuppression with subsequently secondary infections, such as hospital-acquired pneumonia, catheter-associated bacteremia or candidemia, and foley catheter-associated urinary tract infection etc.) usually develop among severe COVID-19 patients who require prolonged invasive ventilation [7, 9]. These problems, in spite of not being unique to COVID-19 patients, are also considered the likely mechanisms thereby significantly increasing the mortality due to the reduction of tolerance of injury in these critically ill patients [7].

The article "Use of Multiple Doses of Intravenous Infusion of Umbilical Cord-Mesenchymal Stem Cells for the Treatment of Adult Patients with Severe COVID-19-Related Acute Respiratory Distress Syndrome: Literature Review" was published in 2023. Journal: Stem Cells Int.

Disappointing outcomes have been shown regarding the therapeutic effect of mesenchymal stem cells (MSCs) for the treatment of influenza pneumonitis [10]. Nevertheless, fetal-like MSCs have been shown to inhibit the activation of M1-type macrophages, as well as elicitation of M2 anti-inflammatory polarization via tumor necrosis factor- (TNF-) *α*-mediated activation of cyclooxygenase-2, and TNF-stimulated gene-6 [11]. An adjuvant treatment using a single dose of intravenous infusion (IVF) of the umbilical cord- (UC-) derived MSCs (UC-MSCs, ranging from 1 × 10^6^ to 10 × 10^6^ cells/kg body weight (kg BW)) was compassionately prescribed to alleviate ARDS seriousness in severe adult COVID-19 patients since 2020, with survival rates reportedly ranging from 50% to 66.7%, while not having any significant adverse effects [12–14]. Despite these results, the clinical effect of multiple-dose IVF-UC-MSCs for the treatment of severe ARDS caused by COVID-19 is undetermined. In 2020, a study conducted by Yip et al. [14] who investigated the efficacy of a single dose of IVF-UC-MSCs at dosages of 1–10 × 10^6^ cells/kg BW for the treatment of nine severe COVID-19 patients with ARDS showed a good result concerning pulmonary function improvement at the initial ARDS stage (see the following text and Table 1).

In 2021, we observed two severe COVID-19 patients (one was a 42-year-old female nurse with morbid obesity (body mass index of 46.7 kg/m^2^), and the other was a 73-year-old male patient with poorly controlled DM) with severe ARDS who received the compassionately salvage IVF-UC-MSCs therapy consisting of multiple doses (four and six cycles since ARDS day (D) 5 (D5), respectively; each MSCs cycle contained 5 × 10^6^ cells/kg BW, kindly provided by the BIONET Corp., Taipei, Taiwan) had the results of successful extubation and survival discharge outcomes (Table 1). Based on the aforementioned experience, we reviewed the relevant PubMed literature database to explore the clinical efficacy of a single-dose or multiple-dose IVF-UC-MSCs for the treatment of COVID-19-induced ARDS among severe COVID-19 patients who received respiratory support of ventilator.

## 2. Materials and Methods

We searched and reviewed the literature from the 2020–2022 PubMed database containing important keywords, including “severe COVID-19,” “ARDS,” “ICU,” “ventilator,” “intravenous administration,” “mesenchymal stromal/stem cells,” “arterial partial pressure of oxygen (PaO_2_),” “fraction of inspired oxygen (FiO_2_),” “pulmonary/lung function,” “survival rates,” “mortality rates” etc.

The article "Use of Multiple Doses of Intravenous Infusion of Umbilical Cord-Mesenchymal Stem Cells for the Treatment of Adult Patients with Severe COVID-19-Related Acute Respiratory Distress Syndrome: Literature Review" was published in 2023. Journal: Stem Cells Int.

## 3. Results

In the review of the PubMed database focusing on the studies investigating the clinical efficacy of multiple-dose IVF-UC-MSCs for the treatment of adult patients with COVID-19-induced ARDS, we found that there were only few surveys recording the detailed data with respect to pulmonary function and the ratios of PaO_2_ to FiO_2_ from the ventilator in severe COVID-19 patients receiving ventilator support. Table 1 summarizes the PubMed literature database regarding the demographic characteristics, various IVF doses of UC-MSCs (predominant adjunctive therapy), and treatment outcomes for adult patients with COVID-19-induced ARDS who received ventilator support in different COVID-19 case series [12–16] with detailed data of PaO_2_/FiO_2_ ratios and the present series.

The Dilogo et al. [12] series enrolling 20 severe COVID-19 patients with ARDS who received therapy of a single IVF-UC-MSCs dose with a dosage of 1.0 × 10^6^ kg BW on an average of post-ARDS 6.5 days showed a case-fatality rate of 50% (10/20), significantly lower than that of those receiving standard care of treatment (80%; *P* = 0.047, using the *χ*^2^ test). Although the differences in the lengths of ICU stay and ventilator usage were not statistically significant between two groups, a rapid improvement in PaO_2_/FiO_2_ ratios was seen among all 10 COVID-19 survivors receiving treatment of a single IVF-UC-MSCs dose (Table 1) [12]. Similar scenarios (also using a single IVF-UC-MSCs dose at the dosage of 1.0 × 10^6^ kg BW) were noted in the Iglesias et al. [13] case series (comprising five COVID-19 patients with severe ARDS, with an in-hospital case-fatality rate of 40% (2/5), as well as the rate of initial improvement in PaO_2_/FiO_2_ ratios of 75% (3/4)) (Table 1). Additionally, a study conducted by Yip et al. [14] compared the difference of efficacy between different single IVF-UC-MSCs dosages [1 × 10^6^ cells/kg BW (*n* = 3), 5 × 10^6^ cells/kg BW (*n* = 3), and 10 × 10^6^ cells/kg BW (*n* = 3)] for the treatment of nine severe COVID-19 patients with ARDS. A single IVF-UC-MSCs dose at the dosage of 10 × 10^6^ cells/kg BW was shown to exhibit the best survival rate (100% (3/3)) among three dosages. Of note, the three MSCs dosages (1–10 × 10^6^ cells/kg BW) resulted in an overall rate of 83.3% (5/6) in lung function improvement among six severe COVID-19 survivors [14]. Furthermore, the Hashemian et al. [15] case series enrolling 11 severe COVID-19 patients who received a three-cycle therapy consisting of 200 × 10^6^ cells/kg BW either IVF-UC- or IVF-placenta-MSCs in each round every other day for alleviating ARDS severity showed an excellent improvement in respiratory function among survivors [100% (8/8)] at the initial treatment stage. However, the D60 survival rate of this series was 54.5% (6/11) [15]. In contrast, Liang et al. [16] also reported a severe COVID-19 case receiving three IVF cycles of 50 × 10^6^ cells/kg BW UC-MSCs every 3 days since ARDS D8 had an improved lung function and a final survival outcome.

The article "Use of Multiple Doses of Intravenous Infusion of Umbilical Cord-Mesenchymal Stem Cells for the Treatment of Adult Patients with Severe COVID-19-Related Acute Respiratory Distress Syndrome: Literature Review" was published in 2023. Journal: Stem Cells Int.

## 4. Discussion

To the best of our knowledge, this is the first review focusing on a full exploration of the efficacy of multiple-dose adjuvant IVF-UC- or placenta-MSCs for treating severe COVID-19-induced ARDS in detail. According to the investigation regarding the biodistribution of IVF-MSCs, the duration of a majority (80%–90%) of IVF-MSCs lodging in the pulmonary vascular bed after administration is short (no more than 48 hr) [17]. Because of a short half-life for IV formulation of MSCs, the receipt frequencies of IVF-UC-MSCs therapy were individually adjusted by us according to the improvement degrees in PaO_2_/FiO_2_ ratios for the two patients at that time. In significant contrast with the Hashemian et al. [15] and the case reported by Liang et al. [16], the two patients cared by us got gradual improvement after the receipt of a prominently lower dosage (5 × 10^6^ cells/kg BW in each infusion) within no more than 5 days of the onset of ARDS [on D4, D10, D15, as well as D18, respectively, for the morbid obesity patient (Table 1); and on D5, D8, D13, D16, D20, as well as D23, respectively, for the diabetic patient (Table 1), not shown in the text]. Despite a considerably lower dosage of MSCs in each cycle prescribed for treatment of these two patients compared to the other two series [15, 16], both two patients finally discharged without sequelae.

A double-blind, randomized controlled trial (RCT) conducted by Monsel et al. [18] who enrolled 21 patients with COVID-19-induced ARDS predominantly receiving three doses of IVF-UC-MSCs (1 × 10^6^ cells/kg BW every other day) showed comparable D28 survival rates (76.2% (16/21) vs. 80% (20/25), *P* = 0.76), but no significant improvement in the change of PaO_2_/FiO_2_ ratios when compared to the placebo group (median, 54.3 vs. 25.3 on D7; *P* = 0.77 as evaluated using analysis of covariance). However, this RCT study did not address the accurate PaO_2_/FiO_2_ data of the patients enrolled in this study [18]. In contrast, an RCT conducted by Lanzoni et al. [19] demonstrated the significant superiority of two adjuvant cycles of IVF-UC-MSCs (100 × 10^6^ cells in each administration, with 72 hr apart) to standard therapy for the treatment of COVID-19-associated ARDS, with mortality rates of 16.7% vs. 58.3% (*P* = 0.035, using the chi-square test) [19]. It is noteworthy that the total dosages of UC-MSCs (5 × 10^6^ cells/kg BW in each infusion; in total of 20–30 × 10^6^ cells/kg BW) prescribed for the treatment of severe ARDS in two severe COVID-19 patients reported by us were higher than those employed in the two aforementioned series [18, 19].

The article "Use of Multiple Doses of Intravenous Infusion of Umbilical Cord-Mesenchymal Stem Cells for the Treatment of Adult Patients with Severe COVID-19-Related Acute Respiratory Distress Syndrome: Literature Review" was published in 2023. Journal: Stem Cells Int.

A review of the PubMed database reveals that a high percentage of severe COVID-19 survivors (including two cases cared by us) with ARDS who received IVF-MSCs on D1–D12 after ARDS onset got a significant improvement of lung function (93.1% (27/29)) before discharge in terms of the PaO_2_/FiO_2_ ratios [12–16]. The excellent clinical efficacy of IVF-UC-MSCs in substantially decreasing the degree of lung dysfunction among severe COVID-19 patients with pneumonitis and ARDS corresponded closely to the surveys of Shi et al. [20] (administering three cycles of 40 × 10^6^ cells every 3 days) and Feng et al. [21] (administering four cycles of 25 × 10^6^ cells every other day). However, a significant diversity in PaO_2_/FiO_2_ levels was still observed among the severe COVID-19 patients enrolled in these two investigations [20, 21].

After SARS-CoV-2 infections, fatal complications besides ARDS (immunosuppression, nosocomial pneumonia, and/or bacteremia, invasive pulmonary aspergillosis and mucormycosis, myocarditis with heart failure, cancer recurrence, pulmonary embolism, and thromboembolism etc.) might subsequently develop in severe COVID-19 patients and adversely affect their outcomes to a considerable degree [22–27]. These complications might plausibly explain the variable survival rates (50%–76%) reported in the five severe COVID-19 case series receiving ventilator support and IVF-MSCs therapy on D1–D16 after the onset of ARDS [12–15, 19].

The limitation of this review article is that many PubMed literature did not accurately record the information regarding the PaO_2_/FiO_2_ ratios and causes of mortality among severe COVID-19 patients with ARDS, and administration days of IVF-UC-MSCs for these patients after the onset of ARDS. Consequently, we could not collect more data for further analysis of the factors compromising the efficacy of IVF-UC-MSCs in improving the case-fatality rates.

## 5. Conclusion

From the aforementioned analyses, the therapy of IVF-UC-MSCs likely improves lung function in severe COVID-19 patients with ARDS, although its role in decreasing mortality rates is usually confounded by various factors (e.g., subsequent septicemic episodes due to the immunosuppressed condition, or thromboembolism caused by SARS-CoV-2 infection etc.). Continued good supportive care is of paramount importance for these critically ill patients. Although the optimal dose, administration frequency, and therapeutic window still need to be investigated by further research, we suggest that the multiple-dose IVF-UC-MSCs at a dosage of 5 × 10^6^ cells/kg BW in each cycle, for at least three rounds (with adjustment of the rounds according to the clinical condition) be considered when determining treatment for severe COVID-19 patients within 5 days of the ARDS onset and before multiorgan failure worsens.

The article "Use of Multiple Doses of Intravenous Infusion of Umbilical Cord-Mesenchymal Stem Cells for the Treatment of Adult Patients with Severe COVID-19-Related Acute Respiratory Distress Syndrome: Literature Review" was published in 2023. Journal: Stem Cells Int.

## Figures and Tables

**Table 1:** Comparison of the demographic characteristics, therapeutic doses of intravenous infusion (IVF) of predominantly umbilical cord (UC) or placenta-harvested mesenchymal stem cells (MSCs), and treatment outcomes among adult patients with COVID-19-induced acute-onset respiratory distress syndrome (ARDS) who received ventilatory support in different severe COVID-19 case series with detailed data regarding ratios of partial pressure in arterial blood oxygen to fraction of inspired oxygen from the ventilator.

References	Single vs. multiple doses of UC-MSCs (number)	Case number (male : female)	Percentage with comorbidities	Dose(s) of UC-MSC cells (case number(s), and administration days after the onset of ARDS)	Ventilator days	Survival rates (%)	Percentage of cases who had a significant improvement in ARDS within 7 days among COVID-19 survivors
Dilogo et al. [12]	Single	20 (15 : 5)	100 (DM, HTN, CKD, CAD, CHF, TB, PPU, obesity, AMI, et al.)	1.0 × 10^6^ kg BW (20; an average of 6.5 days)	15.69 ± 10.37	(In hospital) 50 (10/20)	100 (10/10)
Iglesias et al. [13]	Single	5 (4 : 1)	100 (Obesity, DM, hypothyroidism, HTN, lung fibrosis	1.0 × 10^6^ kg BW (5; D1–D3 after ARDS onset)	1–17	(In hospital) 60 (3/5)	75 (3/4^a^)
Yip et al. [14]	Single	9 (7 : 2)	100 (DM, dyslipidemia, CKD, HTN, recipient of H/D for AKI, liver cirrhosis)	1.0 × 10^6^ kg BW (3; 5–12) 5.0 × 10^6^ kg BW (3; 5–7) 10 × 10^6^ kg BW (3; all were 5) (an average of 6.4 days for overall nine patients)	6–15 15–44 0–8 (an average of 15.4 (±12.9) days)	(In hospital) 66.7 (2/3) 33.3 (1/3) 100 (3/3) (overall 66.7 (6/9))	83.3 (5/6)
Hashemian et al. [15]	Multiple (3 doses, given every other day)	11 (8 : 3)	54.5 (DM, HTN, CLL, CMP)	200 × 10^6^ in each infusion (6 received UC-MSCs, while 5 received placental MSCs; at medians of D5, D7, and D9, respectively, after ARDS onset)	An average of 3, among 7 patients who had initial improvement	(D60) 54.5 (6/11)	100 (8/8^b^)
Liang et al. [16]	Multiple (3 doses, 72 hr apart)	1 (0 : 1)	0	50 × 10^6^ in each infusion (1; D8, D11, and D14, respectively, after onset of ARDS)	12	(D30) 100 (1/1)	100 (1/1)
Jean et al. (authors' series)	Multiple (4–6 doses)	2 (1 : 1)	100 ((Case 1) Morbid obesity, and (case 2) DM, respectively)	5 × 10^6^ kg BW in each infusion (2; for case 1, 4 doses: on D4, D10, D15, and D18; for case 2, 6 doses: on D5, D8, D13, D16, D20, and D23, respectively, after ARDS onset)	28 and 46, respectively	(In hospital) 100 (2/2)	100 (2/2)

UC-MSCs, umbilical cord of mesenchymal stem cells; M : F, male : female; ARDS, acute-onset respiratory distress syndrome; DM, diabetes mellitus; HTN, hypertension; CKD, chronic kidney disease; H/D, hemodialysis; AKI, acute kidney injury; BW, body weight; CAD, coronary artery disease; CHF, congestive heart failure; TB, *Mycobacterium tuberculosis* infection; PPU, perforated peptic ulcer; AMI, acute myocardial infarction; D, days; Afib, atrial fibrillation; CVA, cerebrovascular accident; CLL, chronic lymphocytic lymphoma; CMP, cardiomyopathy; NA, not applicable. ^a^One patient died on Day 15 after IV UC-MSCs infusion due to bacterial pneumonia and hepatic failure with active bleeding. ^b^One patient received the first dose of IVF-MSCs on Day 11 of admission of intensive care unit (ICU). A definite improvement in the pulmonary dysfunction was initially noticed, but this patient died due to sudden-onset cardiac arrest (unrelated to MSC infusion) 4 days after this IVF-MSCs dosing. The other patient, who received the first dose of IVF-MSCs on ICU admission Day 5, had a similar clinical scenario.

The article "Use of Multiple Doses of Intravenous Infusion of Umbilical Cord-Mesenchymal Stem Cells for the Treatment of Adult Patients with Severe COVID-19-Related Acute Respiratory Distress Syndrome: Literature Review" was published in 2023. Journal: Stem Cells Int.

## Data Availability

The data used to support the conclusions of this investigation are added in this article.

## Abbreviations

SARS-CoV-2: Severe respiratory syndrome coronavirus 2
COVID-19: Coronavirus disease 2019
ARDS: Acute respiratory distress syndrome
DM: Diabetes mellitus
ICU: Intensive care unit
MSCs: Mesenchymal stem cells
IVF: Intravenous infusion
UC: Umbilical cord
D: Day
PaO_2_: Arterial partial pressure of oxygen
FiO_2_: Fraction of inspired oxygen
RCT: Randomized controlled trial.
